RETRACTED

# A Cohort Study on the Safety and Efficacy of Warfarin and Rivaroxaban in Anticoagulant Therapy in Patients with Atrial Fibrillation Study

**DOI:** 10.1155/2022/4611383

**Published:** 2022-07-07

**Authors:** Li Wang, Wentao Yao

**Affiliations:** Department of Pharmacy, Anji People's Hospital, Huzhou City, Zhejiang, Province 313300, China

## Abstract

**Objective:**

To observe the safety and efficacy of warfarin and rivaroxaban in anticoagulation therapy in patients with atrial fibrillation (AF).

**Methods:**

A total of 96 patients with AF treated in our hospital from June 2019 to February 2021 were enrolled in this study. According to the different modes of drug administration, the patients were divided into the warfarin group and rivaroxaban group. Demographic and clinical data such as age, body weight, and previous drug use were collected. The blood routine, liver and kidney function, blood coagulation routine, and cardiac color ultrasound were accessed. The valvular atrial fibrillation and anticoagulant taboos were excluded, and the risk of embolism and bleeding was evaluated. Among them, 48 patients in the warfarin group were given warfarin once a day, and the international ratio (INR) was used to adjust the dose, and the INR was controlled between 2.0 and 3.0. In contrast, 48 patients in the rivaroxaban group received a fixed dose of rivaroxaban 20 mg or 15 mg once a day. After administration, regular telephone or outpatient follow-up was given once a month, to monitor patients' drug compliance and ask if there was bleeding, and to detect blood routine, urine routine, fecal routine+occult blood, and liver and kidney function. In addition, at the beginning of 3, 6, and 12 months of follow-up, each patient was given cardiac color Doppler ultrasound, peripheral vascular color ultrasound, and brain CT to determine whether there were mural thrombosis, stroke, and peripheral arterial thromboembolism. The INR attainment rate, coagulation index, thromboembolism, bleeding, and adverse reactions were compared between the two groups.

**Results:**

There was no significant difference in serum Dmurd and NT-proBNP levels between the two groups before treatment and 3, 6, and 9 months after treatment. There was no significant difference in the number of venous embolism, pulmonary embolism, cerebral embolism, and total embolism between the two groups (*P* > 0.05). There was no significant difference in the number of mild, moderate, and severe bleeding between the two groups (*P* > 0.05), but the total number of bleeding in the rivaroxaban group was lower than that in the warfarin group (*P* < 0.05). During the treatment, side effects such as nausea and vomiting, elevated transaminase, glutamyl transpeptidase, and diarrhea occurred between the two groups, and there was no significant difference in the number of adverse reactions between the two groups (*P* > 0.05).

RETRACTED

**Conclusion:**

Compared with warfarin, rivaroxaban anticoagulant therapy has the same advantage in tolerance and prevention of thromboembolism in patients with AF, but rivaroxaban can effectively reduce the risk of bleeding in patients with AF.

## 1. Introduction

Atrial fibrillation (AF) remains one of the most common and serious arrhythmias in clinic, and it is a difficult problem in the world that modern medicine urgently needs to overcome [1]. In recent years, the number of patients with AF is increasing, and the morbidity and mortality are also increasing year by year. AF is easy to cause a variety of complications, which is the leading cause of stroke, and it is prone to lead to death and disability. Moreover, the stroke incidence of patients with AF is five times higher than that of normal people [2]. In addition, atrial fibrillation is an independent risk factor for stroke. Atrial fibrillation not only causes coronary heart disease and is closely related to the death of patients with coronary heart disease but also promotes the occurrence of stroke [3]. The CHADS2 scoring system was proposed in 2006 guidelines for the diagnosis and treatment of atrial fibrillation [4]. In this scoring system, hypertension, heart failure, and diabetes are independent risk factors for stroke in patients with AF with a score of 1 for each item. If the patient had a history of stroke, TIA, or thrombosis, the score was twice as high as that of other risk factors. When the CHADS score of patients with AF is ≥2, the incidence of stroke is higher, so it is necessary to standardize the use of anticoagulants [4]. Various risk factors must be scored strictly according to the guidelines for the diagnosis and treatment of AF, the risk of stroke must be strictly assessed, and anticoagulant therapy should be given to patients with AF in time.

In the anticoagulant therapy of AF, traditional anticoagulants are used before the emergence of new anticoagulants and play an indispensable role. Warfarin is the most widely used traditional anticoagulant in clinic. It is a kind of coumarin anticoagulant, which can inhibit thrombosis in vivo by inhibiting the synthesis of coagulation factors involved in vitamin K in the liver [5]. Warfarin is a widely used anticoagulant in clinic, but it also has some shortcomings. For example, the treatment window is narrow; coagulation INR needs to be monitored regularly; it is inconvenient for out-of-hospital patients to adjust dose, individual dose difference, high risk of bleeding, easy to be affected by food and drugs, and so on, which make clinical anticoagulation therapy relatively complex; and patient compliance and drug efficacy are not good [6]. Many patients with anticoagulant guidelines only use antiplatelet therapy or even no treatment due to difficulties in INR control and concerns about the risk of bleeding. Nowadays, new oral anticoagulants have been gradually developed. Until 2010, direct thrombin inhibitor dabigazone was approved by FDA for thromboembolism prevention in patients with atrial fibrillation [7]. Subsequently, Xa factor inhibitors rivaroxaban and apixaban were also approved for thrombosis prevention after orthopedic surgery. Dabigatran and rivaroxaban can be used in the treatment of venous thrombosis [7–9]. Rivaroxaban is the representative drug of Xa factor inhibitor, and its mechanism is a Xa factor inhibitor into the body, can specifically directly inhibit Xa factor, can combine with free, and bound Xa factor to play a role. Subsequently, it blocks the conversion of prothrombin (factorII) to thrombin (Ia factor), inhibits the production of thrombin, and achieves the effect of anticoagulation and prevention and treatment of thrombus [8]. It is worth noting that some studies have proposed that the procoagulant effect of Xa factor is relatively simple, but the role of thrombin is more complex, and continuous inhibition of it may lead to abnormal hemostatic regulation, while Xa factor inhibitors will not affect normal hemostasis [10]. In this study, the efficacy and safety of new anticoagulant rivaroxaban and traditional anticoagulant warfarin were observed and analyzed. Then, the efficacy and safety of new anticoagulants in patients with atrial fibrillation were discussed in order to provide reference basis for clinical diagnosis and provide certain guiding significance for clinical medication in the future. The results are reported as follows.

RETRACTED

## 2. Patients and Methods

### 2.1. Patient Information

A total of 96 patients with AF treated in our hospital from June 2019 to February 2021 were selected. According to the different modes of drug administration, the patients were divided into the warfarin group (*n* = 48) and rivaroxaban group (*n* = 48). Inclusion criteria are as follows: (1) according to June 2014, the National Institute of Health and Clinical Optimization (NICE) issued a new atrial fibrillation management guide based on the 2006 edition of the Atrial Fibrillation Management Guide [11]: patients who meet the diagnostic criteria of atrial fibrillation. Atrial fibrillation can be diagnosed if the following three items are satisfied: (1) the electrocardiogram shows that the absolute RR interval is different; (2) there is no obvious wave in ECG, but relatively regular atrial electrical activity can also be seen in some leads (the most common lead is V, lead); and (3) the interval between two atrial electrical activities usually changes, and the time limit is generally less than 200 ms. Paroxysmal atrial fibrillation means that atrial fibrillation can be recovered by itself or with intervention within 7 days. Persistent atrial fibrillation means atrial fibrillation lasts for more than 7 days. Nonvalvular atrial fibrillation refers to (1) atrial fibrillation with no rheumatic mitral stenosis, no mechanical or biological valve, and no history of mitral valve repair; (2)18 years old ≤ age ≤ 75 years old; (3) male CHA2DS2-VAScscore ≥ 2, female CHA2DS2-VAScscore ≥ 3 0; (4) HAS-BLEDscore < 3[12]; (5) good medication compliance, can accept long-term follow-up, and actively cooperate with related treatment and examination; (6)body mass index (BMI) < 30 kg; (7) basic diseases (such as diabetes and hypertension) before entering the group have been effectively controlled; (8) there are no anticoagulation contraindications (such as severe hepatic and renal insufficiency, severe hypertension (≥180/110 mmHg), history of blood disease or digestive tract ulcer, etc.); and (9) the patients and their families have informed consent.

Exclusion criteria are as follows: (1) there were ischemic stroke and operation in recent 3 months and history of trauma or combination of nonsteroidal anti-inflammatory drugs and antiplatelet drugs; (2) allergic constitution or allergy to drugs used in this study; (3) alcoholism, history of artificial heart valve replacement or history of deep venous thrombosis, cerebral hemorrhage, pulmonary embolism, and rheumatic heart disease; (4) patients with malignant tumor, thrombocytopenia, or hemorrhagic disease; (5) patients with history of urinary or digestive system bleeding within one year; (6) severe hepatic insufficiency and renal insufficiency (Child-Pugh grade B and C, creatinine clearance < 30 mL/min). Creatinine clearance rate (Cer) was calculated by Cockcroft-Gault equation: male Ccr (mL/min) = [140 − age (age)] × body mass (kg)/[72 × serum creatinine (mg/dL)], female Ccr (mL/min) = 0.85 × [140 − age (age)] × body mass (kg)/[72 × serum creatinine (mg/dL)], which results in normal range values as follows: adults 80~12 mL/min; and (7) patients who did not follow the doctor's advice or missing cases.

### 2.2. Treatment Method

All patients were treated with the same ventricular rate and rhythm control, and the specific medication plan can be referred to recommendation. It mainly includes (1) compartment rate control: commonly used drugs include amiodarone, digitalis (such as digoxin and lanoside C), *β*-blockers (such as metoprolol, atenolol, and bisoprolol), etc. 2 rhythm control: cardioversion of rapid atrial fibrillation: commonly used drugs include amiodarone, ibutilide, propafenone, etc. Long-term treatment to maintain sinus rhythm: there are Xenedarone, sotalol, amiodarone, and other drugs.

RETRACTED

The warfarin group is as follows: (1) on this basis, antithrombotic therapy was given to warfarin (Shanghai Xinyi Pharmaceutical Factory, Chinese medicine H31022123); specifically, the initial dose was 2.5 mg/d, and the coagulation index was monitored for 1 time before treatment, and the international standardized ratio (INR) value was determined. (2) After 3 days, 6 days, and 9 days of treatment, the INR value was rechecked, and the INR value was timely adjusted according to the dose of warfarin. (3) If the INR value reaches 1.6 to 2.5 for two consecutive times, the frequency of INR can be adjusted to once a week, and if it is stable for another two weeks, it can be adjusted to the first month. (4) If the INR value is outside the target range for two consecutive times, the dose of warfarin should be adjusted in time, and the monitoring of blood coagulation index should be strengthened. (5) The specific ways to deal with bleeding complications and the increase of INR value during medication are as follows. INR > 3.0: 4.5 (no bleeding complications): actively analyze and deal with the causes of abnormal INR. If it is caused by drug overdose, reduce the original dose by 5% to 20% or stop taking it once. Monitor the INR after 1-2 days, adjust the dose according to the INR value until the INR reaches the standard, and strengthen INR monitoring in the later stage. INR > 4.5 ~ <10.0 (no bleeding complications): the use of anticoagulants was suspended and the corresponding hemostatic drugs were used. INR was measured after 6 hours and 12 hours. Start warfarin therapy with 2.5 mg once a day until INR < 3. INR ≥ 10.0 or severe bleeding (regardless of INR level): stop using anticoagulant warfarin and actively use corresponding hemostatic drugs. After the condition is stable, we will determine whether to continue to use warfarin according to the analysis of the causes of bleeding.

The rivaroxaban group is as follows: on the basis of the above ventricular rate and rhythm control therapy, the patients in the experimental group were treated with rivaroxaban (German Bayer Schering Pharmaceutical, approval no. H20140132). According to the Chinese consensus of rivaroxaban, the dosage was determined according to the creatinine clearance rate (Ccr), age and body weight of the patients, taking 20 mg/days when Ccr ≥ 50 mL/min and 15 mg/days when Ccr was 30-49 mL/min. Chew and take it with the food at the same time during the meal. If you miss it, make it up within 12 hours. If it is more than 12 hours, you do not need to take it. If you forget whether to take the drug or not during the period of taking it, you can take it once. If you take double dose, continue to take the next drug according to the original plan. If bleeding occurs during medication, it is recommended to seek medical treatment in time to promote drug excretion, hemostasis, and other treatment. Meanwhile, in order to effectively improve the compliance of each patient with long-term medication, we should strengthen the knowledge education and evaluate the cognitive function of patients with AF before treatment.

RETRACTED

### 2.3. Observation Index

Embolism events are as follows: the occurrence of venous embolism, pulmonary embolism, and cerebral embolism of lower extremities during the treatment of the two groups were recorded in detail. Bleeding events are as follows: record in detail the spontaneous bleeding events of all patients during medication, including (1) slight bleeding, such as microscopic hematuria, conjunctival or skin bleeding, nasal worms, blood in sputum, ecchymosis, and gingival bleeding, or the decrease of hematocrit (HCT) < 9%, or the decrease of hemoglobin (Hb) < 30 g/L. (2) A small amount of bleeding: if there are black stool or bloody stool, a small amount of hematemesis or hemoptysis, gross hematuria, or 10% ≤ HCT decrease <15%, or 30 g/L ≤ Hb drop < 50 g 300 mL. (3) Severe hemorrhage: if there is cerebral hemorrhage, or blood transfusion > 400 mL, one time bleeding volume ≥ 300 mL, or massive extracranial hemorrhage such as massive hemoptysis and gastrointestinal hemorrhage, or HCT decrease ≥ 15%, or Hb decrease ≥ 50 g/L. Detection of plasma indexes are as follows: (1) fasting elbow venous blood was taken from each patient before treatment and 3 and 6 months after treatment, 3 mL/times, and plasma was separated by centrifugation and stored in refrigerator at -20°C to be tested. (2) The instrument selected automatic enzyme labeling instrument (Shandong Boko, model BIOBASE-EL10A), and INR and D-DNT-proBNP were determined by enzyme-linked immunosorbent assay (ELISA). (3) The kits are all purchased from Shanghai Jianglai Biology, and the above index detection steps are carried out strictly according to its supporting instructions.

Adverse reactions are as follows: the adverse reactions/events caused by drugs in the two groups were recorded in detail, such as dizziness and headache, elevated transaminase, diarrhea, and other adverse reactions/events.

RETRACTED

### 2.4. Statistical Analysis

SPSS 21.0 statistical software is used to analyze the normal distribution and homogeneity of variance of the measurement data before statistical analysis, which meets the requirements of normal distribution or approximate normal distribution. The variance of repeated measurement data is expressed as $\bar{x}\pm s$. *T*-test was used to compare the two groups, *n* (%) was used to represent the counting data, and *χ*^2^ test was used. When *P* < 0.05, the difference was statistically significant.

## 3. Results

### 3.1. Comparison of General Clinical Data between the Two Groups

There was no significant difference in sex, age, body mass index, creatinine, creatinine clearance rate, basic disease history, CHA2DS2-VASc score, and HAS-BLED score between the warfarin group and rivaroxaban group. The two groups of patients are comparable (*P* > 0.05). All the results are presented in Table 1.

### 3.2. The Plasma Indexes of the Two Groups Were Compared in Each Time Period

There was no significant difference in serum Dmurd and NT-proBNP levels between the two groups before treatment, 3 months after treatment, 6 months after treatment, and 9 months after treatment (*P* > 0.05). All the results are presented in Table 2.

### 3.3. Comparison of Embolism between the Two Groups

There was no significant difference in the number of venous embolism, pulmonary embolism, cerebral embolism, and total embolism between the two groups (*P* > 0.05). All the results are presented in Table 3.

### 3.4. Comparison of Bleeding between the Two Groups

There was no significant difference in the number of mild, moderate, and severe bleeding between the two groups (*P* > 0.05), but the total number of bleedings in the rivaroxaban group was significantly lower than that in the warfarin group (*P* < 0.05). All the results are presented in Table 4.

### 3.5. The Levels of Serum NSE and MBP Were Compared between the Two Groups at 1 Day before Operation, 1 Day after Operation, 3 Days after Operation, and 7 Days after Operation

During the treatment, adverse reactions such as nausea and vomiting, elevated transaminase, glutamyl transpeptidase, and diarrhea occurred in the two groups, but there was no significant difference in the number of adverse reactions between the two groups (*P* > 0.05). All the results are presented in Table 5.

## 4. Discussion

AF is one of the most common and serious arrhythmias in clinic, which is a difficult problem in the world that modern medicine urgently needs to overcome. Many scholars have surveyed the etiology, pathogenesis, treatment, clinical manifestations, and complications of atrial fibrillation [3]. Zhiqiang and scholars have conducted large-scale epidemiological investigations on patients with AF in 13 provinces of China. The study indicates that the prevalence rate of AF in China is 0.77%. The prevalence rate of AF in males (0.9%) is slightly higher than in females (0.7%), and there is a tendency to increase with age [13]. It should be noted that atrial fibrillation is prone to more complications. Patients with atrial fibrillation are the primary cause of stroke, which is easy to be killed and disabled, and the consequences will be very serious, which will not only bring heavy family burden to patients and their families but also bring considerable difficulties to the treatment of clinicians [12]. Therefore, the treatment of AF has attracted great attention all over the world. The incidence of stroke in AF patients is 5 times higher than that in normal subjects [14]. Its clinical manifestations are chest tightness, shortness of breath, dizziness, palpitation, and so on. When AF occurs, the heartbeat is fast and irregular, resulting in the loss of effective contraction of the atrium and ventricle, resulting in a decrease in cardiac output and a hemodynamic disorder [11].

RETRACTED

The complications of AF are very serious, and the national consciousness should be strengthened. When there are similar clinical manifestations of AF, we should pay close attention to whether the disease is AF and go to the hospital in time, so as to prevent the occurrence of complications of AF. Therefore, active treatment should be taken during the attack of AF to avoid the occurrence of complications [8]. In recent years, the number of patients with AF is increasing, and the morbidity and mortality have been paid more attention. The independent risk factors associated with AF include advanced age, diabetes, myocardial infarction, heart failure, and valvular heart disease [15]. Cardiomyopathy, hypertensive heart disease, heart failure, rheumatic heart disease, cardiac surgery, preexcitation syndrome, sick sinus syndrome, hyperthyroidism, and infection are closely related to the occurrence of AF [15]. Therefore, patients with independent factors related to AF should be paid close attention to avoid the occurrence of AF and the occurrence of complications of AF, in order to reduce the rate of death and disability. So far, the pathogenesis of AF has not been fully elucidated. The pathogenesis of AF may be closely related to the anatomical structure of the atrium, atrial electrophysiology, and arrhythmia. Therefore, understanding the anatomical structure of atrium, atrial electrophysiology, and the mechanism of arrhythmia is helpful to understand the pathogenesis of AF. Some studies have shown that the prolongation of atrial refractory period can induce the occurrence of AF [15]. Only by understanding the anatomical structure of the atrium, the electrophysiology of the atrium, and the mechanism of arrhythmia can we better understand the pathogenesis of atrial fibrillation, prevent the occurrence of atrial fibrillation, avoid the complications of atrial fibrillation, and reduce the risk of anticoagulation therapy. AF is beneficial and reduces the risk of AF complications [15].

RETRACTED

When the attack of AF lasts for more than 48 hours, it is very easy to form mural thrombus in the heart [16]. At present, it is considered that there are three main factors leading to thrombosis induced by AF: injury of cardiac endothelium, hemodynamic changes, and abnormal blood composition [17]. In patients with AF, atrial dilatation, decreased contractile function, cardiac valve stenosis, or insufficiency led to changes in cardiac hemodynamics, prone to form blood stasis and turbulence, increase the contact between platelets and cardiac endothelium, and increase the chance of platelet activation, and stagnant blood flow will increase the concentration of thrombin in the local blood flow of the heart and lead to thrombus [17]. On the other hand, atrial stunning and the decrease of contractile function of the left atrium and left atrial appendage will lead to the decrease of local shear stress of the atrium and atrial appendage, which in turn leads to the decrease of nitric oxide and thrombus. Some scholars have confirmed that there is endothelial injury in patients with AF, endothelial injury leads to the decrease of blood eNOS activity and expression, coupled with the increase of von Willebrand factor and endogenous anticoagulant molecules increase the risk of thrombosis. In addition, the activation of the coagulation system and fibrinolysis system in blood decreased, and platelet self-activation and inflammation also increased thrombosis in patients with atrial fibrillation [18]. When the heart mural thrombus forms and falls off with the blood flow to various tissues, it will cause cerebral embolism and extracranial thromboembolism. Cerebral embolism caused by atrial fibrillation is also known as cardiogenic stroke. At present, it is clear that AF is an important influencing factor of embolic stroke. According to related research data, AF can increase the incidence of stroke by 6-8 times. Patients with AF not only have a higher risk of stroke than those without AF but also have a greater risk of stroke than those caused by other causes [19]. Studies have shown that stroke mortality in patients with AF is as high as 20%, and the disability rate is about 60% [20].

RETRACTED

According to the 2019 atrial fibrillation guidelines revised by the American Heart Association, the American College of Cardiology, and the European Heart Association, all patients with AF who meet the criteria for anticoagulant use should use anticoagulants to prevent thrombosis through clinical characteristics such as sex, age, high blood pressure, and heart disease risk, except for isolated atrial fibrillation or contraindications [21]. The 2010 ESC guidelines for the diagnosis and treatment of AF clearly state that if the CHA-DS-VASc score is ≥2, patients are advised to take anticoagulant therapy and long-term anticoagulant therapy [22]. Warfarin is the most widely used traditional anticoagulant in clinic. It plays an important role in the history of the treatment of AF. It is a kind of coumarin anticoagulant, which has a certain anticoagulant effect on the treatment of AF before the emergence of new anticoagulants. It can inhibit thrombosis in vivo by inhibiting the synthesis of coagulation factors involved in vitamin K in the liver. The use of warfarin reduces the incidence of stroke, and the effective dose of warfarin varies due to individual differences, which results in the need to draw blood to detect the international standardized ratio (INR) [23] in the use of warfarin in order to adjust the dosage of warfarin. This tedious treatment process reduces the antithrombotic effect of warfarin to some extent. Because of its narrow treatment window, large individual differences in dose response, relatively high risk of hemorrhage, and the interaction between Chinese farin and food or drugs during treatment, the incidence of cerebral hemorrhage in elderly patients and patients with renal insufficiency increased. As a result, the clinical benefit is greatly reduced. Therefore, after the emergence of new anticoagulants, the utilization rate of anticoagulant effect of warfarin in the treatment of atrial fibrillation has been greatly reduced. Rivaroxaban is a highly selective oral inhibitor that can directly inhibit Xa factor and plays an important role in anticoagulation. It acts on blocking endogenous and exogenous blood coagulation pathways, so as to achieve the purpose of anticoagulation and inhibition of thrombus. Rivaroxaban has the advantages of safety, effectiveness, and convenience in the prevention and treatment of thromboembolic diseases [23]. In many clinical studies, the efficacy of rivaroxaban in preventing stroke in patients with atrial fibrillation is not significantly different from that of warfarin, but it can effectively improve anticoagulant effect, significantly reduce the occurrence of severe bleeding events, and reduce the pain of patients [24, 25]. In this study, the efficacy and safety of new anticoagulant rivaroxaban and traditional anticoagulant warfarin in the treatment of AF were observed and analyzed, and the efficacy and safety of new anticoagulant in patients with AF were discussed, in order to provide a reference basis for clinical diagnosis and provide a certain guiding significance for the clinical use of drugs in the future.

RETRACTED

The results showed that there was no significant difference in serum D-D and NT-proBNP levels between the two groups before treatment and 3, 6, and 9 months after treatment. It shows that warfarin anticoagulation therapy and rivaroxaban anticoagulation therapy can achieve better anticoagulation effect in patients with AF. D-D is a specific degradation product, which can effectively reflect the function of fibrinolysis. When there are fibrinolytic activity and activated thrombosis in the blood vessels, the content of D-D will increase significantly. Meanwhile, the patients with diffuse intravascular coagulation (DIC), pulmonary embolism (PE), deep venous thrombosis (DVT), and other pathological conditions can also cause the increase of D-D level. Some literatures have shown that there is a certain degree of hypercoagulable state in patients with AF, and the content of D-D can be used as an important reference index to evaluate the risk of embolism in patients with AF [26]. NT-proBNP is an objective marker for clinical evaluation of cardiac function. When patients present with AF, it can cause changes in ventricular volume and increase in atrial pressure, resulting in a large number of synthesis and secretion of NT-proBNP. In addition, atrial myocytes are very easy to induce degenerative fibrosis during persistent AF, which further promotes the release of NT-proBNP by cardiomyocytes (CMC) and then damages the endothelial function and increases blood concentration and viscosity, which indirectly leads to thrombosis. Therefore, monitoring the level of NT-proBNP is of great significance in judging the prethrombotic state in patients with AF. The results of this study showed that compared with those before treatment, the plasma levels of D-D and NT-proBNP in the two groups were gradually improved after 3, 6, and 9 months of treatment, but there was no significant difference between the rivaroxaban and warfarin at 3, 6, and 9 months after treatment, which suggested that antithrombotic therapy with the above two drugs could effectively improve the blood hypercoagulable state and reduce the risk of embolism in patients with AF. This is consistent with the occurrence of thromboembolic events in the two groups in this study. The results of this study suggested that lower limb venous embolism, pulmonary embolism, and cerebral embolism occurred in both groups during the treatment period, but there was no significant difference in the number of embolism events and total embolism cases between the two groups (*P* > 0.05).

RETRACTED

Warfarin is a medium-acting anticoagulant, and its mechanism and advantages in the treatment of AF are as follows: (1) through competitive antagonism to vitamin K (VitK), block the synthesis of coagulation factor IX by hepatocytes and then play an anticoagulant effect; (2) reduce platelet aggregation rate (PAR) by inhibiting thrombin (Thr) activity and then play the role of anti-platelet aggregation (PA); (3) high bioavailability; and (4) it can effectively inhibit the occurrence of embolism and the shedding of thrombus, prevent the extension and expansion of thrombus, and inhibit the formation of new thrombus. However, there are still many limitations in clinical use. For example, it is easy to interact with a variety of drugs and foods; sometimes, it needs heparin, narrow treatment window, and metabolic gene polymorphism and needs laboratory monitoring of blood coagulation indicators to adjust drug dosage, slow effect, and so on. Thus, it can be seen that it is far from enough for patients with atrial fibrillation to rely solely on warfarin for anticoagulant therapy.

Rivaroxaban is a coagulation factor Xa (FXa) inhibitor. The main mechanism of its anticoagulation is that it directly and selectively inhibits FXa, which interrupts the exogenous and endogenous pathway of coagulation waterfall and then inhibits the formation of FXa. It can block the cascade amplification effect mediated by FXa and play an anticoagulant effect [22]. The advantages of rivaroxaban are (1) small molecular weight and almost insoluble in water; (2) oral absorption is not affected by food and takes effect quickly; (3) it has little effect on the existing Thr activity, so it has little effect on physiological hemostatic function; (4) it takes a single coagulation factor as the target, so there are few kinds of drugs that can affect its efficacy; and (5) there is no need to monitor INR frequently during treatment. Studies have shown that rivaroxaban in patients with AF is safe and effective and can significantly shorten the time of cardioversion. A meta-analysis also shows that rivaroxaban therapy in patients with AF has high efficacy and safety and can significantly reduce stroke, intracranial hemorrhage, and mortality [27]. The ROCKETAF trial indicates that rivaroxaban has a potential advantage as an alternative to warfarin in the prevention of systemic embolism and stroke in patients with atrial fibrillation [27]. Of note, it is recommended that elderly patients with AF who are unstable in INR, bleed with warfarin in the past, and are unwilling or unable to receive warfarin treatment should give priority to drugs such as rivaroxaban and dabigatran [27].

RETRACTED

Researches have unveiled that most patients with AF are complicated with thrombosis. In this study, the incidence of thrombosis in patients with AF treated with rivaroxaban and warfarin for 9 months was only 6.25% and 8.33%, respectively, and there was no significant difference between the two groups. It is suggested that the effects of the above two drugs in preventing thromboembolic events in patients with AF are similar, which is consistent with the reported results [16]. Our current study shows that the incidence of bleeding within 9 months in the rivaroxaban group is significantly lower than that in the warfarin group, indicating that rivaroxaban treatment is more beneficial to reduce bleeding events and reduce the degree of bleeding in patients with atrial fibrillation. From the point of view of adverse drug reactions, the side effects of the two groups were mainly concentrated in the nervous system and gastrointestinal tract, but the symptoms were mild and no other serious events were found, and there was no significant difference in the total incidence of adverse reactions between the two groups. It can be seen that patients with AF have high tolerance to the above two drugs.

Conclusively, compared with warfarin, rivaroxaban has the same advantages in tolerance and prevention of thromboembolism in patients with atrial fibrillation, but rivaroxaban can more effectively reduce the risk of bleeding in patients with atrial fibrillation. However, there are still some problems in this study, such as incomplete observation index, short follow-up time, and limited sample size, which need to be further demonstrated and analyzed by more prospective, large-sample, multicenter randomized controlled trials.

## Figures and Tables

**Table 1:** Comparison of general clinical data between the two groups (*n* (%), $\bar{x}\pm s$).

Data	*n*	Warfarin formation (*n* = 48)	Rivaroxaban formation (n =48)	*χ* ^2^/*t*	*P*
Gender					
Male	45	20 (44.44)	25 (55.56)		
Female	51	28 (54.90)	23 (45.10)	1.045	0.306
Age (year)	96	58.32 ± 10.25	56.79 ± 11.21	0.697	0.487
Body mass index (kg/m^2^)	96	25.86 ± 2.25	25.63 ± 2.35	0.489	0.625
Serum creatinine (umol/L)	96	77.56 ± 11.72	80.63 ± 12.66	1.232	0.220
Creatinine clearance rate(mL/min)	96	57.34 ± 13.02	58.16 ± 13.56	0.302	0.763
High blood pressure					
Yes	52	28 (53.85)	24 (46.15)		
No	44	20 (45.45)	24 (54.56)	0.671	0.412
Diabetes					
Yes	39	18 (46.15)	21 (53.85)		
No	57	30 (52.63)	27 (47.37)	0.388	0.533
Smoking					
Yes	47	22 (46.81)	25 (53.19)		
No	49	26 (53.06)	23 (46.94)	0.375	0.540
Drink alcohol					
Yes	36	19 (52.78)	17 (47.22)		
No	60	29 (48.33)	31 (51.67)	0.177	0.673
Heart failure					
Yes	22	12 (54.55)	10 (45.45)		
No	74	36 (48.65)	38 (51.35)	0.235	0.627
CHA2DS2-VASc scoring	96	3.19 ± 0.72	3.38 ± 0.88	1.157	0.249
HAS-BLED scoring	96	2.27 ± 0.44	2.18 ± 0.35	1.109	0.270

RETRACTED

**Table 2:** Comparison of serum Dmurd and NT-proBNP levels in different time periods between the two groups $\bar{x}\pm s$.

Group	*N*	D-D ($\bar{x}\pm s$, ng/mL)				NT-proBNP ($\bar{x}\pm s$, pg/mL)			
		Before treatment	3 months after treatment	6 months after treatment	9 months after treatment	Before treatment	3 months after treatment	6 months after treatment	9 months after treatment
Warfarin formation	48	357.12 ± 61.83	214.42 ± 32.58^a^	112.17 ± 22.16^a^	108.76 ± 21.25^a^	3151.38 ± 354.53	1931.42 ± 316.15^a^	723.84 ± 125.45^a^	701.87 ± 124.53^a^
Lifashaban formation	48	366.97 ± 56.64	219.84 ± 33.22^a^	115.18 ± 24.81^a^	110.85 ± 22.03^a^	3018.89 ± 362.24	1839.61 ± 322.76^a^	753.92 ± 136.47^a^	728.27 ± 135.38^a^
*t*		0.813	0.807	0.626	0.473	1.811	1.407	1.124	0.994
*P*		0.417	0.421	0.532	0.637	0.073	0.162	0.263	0.322

Note: compared with that before treatment, ^a^*P* < 0.05 in this group.

**Table 3:** Comparison of embolism between the two groups (*n*, %).

Group	*N*	Lower extremity venous embolism	Pulmonary embolism	Cerebral embolism	Total number of embolism cases
Warfarin formation	48	2 (4.17)	1 (2.08)	1 (2.08)	4 (8.33)
Lifashaban formation	48	1 (2.08)	1 (2.08)	1 (2.08)	3 (6.25)
*χ* ^2^		0.344	0.000	0.000	0.154
*P*		0.557	1	1	0.694

**Table 4:** Comparison of thrombus bleeding between the two groups (*n*, %).

Group	*N*	Slight bleeding	Moderate bleeding	Severe bleeding	Total number of bleeding cases
Warfarin formation	48	6 (12.50)	3 (6.25)	1 (2.08)	10 (20.83)
Lifashaban formation	48	2 (4.17)	1 (2.08)	0 (0.00)	3 (6.25)
*χ* ^2^		2.181	1.043	1.010	4.359
*P*		0.139	0.307	0.314	0.036

Note: compared with the control group, ^a^*P* < 0.05.

**Table 5:** Comparison of adverse reactions between the two groups (*n*, %).

Group	*N*	Nausea and vomiting	Elevated transaminase	Glutamyl transpeptidase	Diarrhea	Total number of adverse reactions
Warfarin formation	48	2 (4.17)	1 (2.08)	3 (6.25)	2 (4.17)	8 (16.67)
Lifashaban formation	48	2 (4.17)	2 (4.17)	2 (4.17)	1 (2.08)	7 (14.58)
*χ* ^2^		0.000	0.344	0.211	0.344	0.079
*P*		1	0.557	0.645	0.557	0.778

## Data Availability

No data were used to support this study.
